The article "LSM-SEC: Tongue Segmentation by the Level Set Model with Symmetry and Edge Constraints" was published in 2021. Journal: Comput Intell Neurosci.

# LSM-SEC: Tongue Segmentation by the Level Set Model with Symmetry and Edge Constraints

**DOI:** 10.1155/2021/6370526

**Published:** 2021-07-29

**Authors:** Shanshan Gao, Ningning Guo, Deqian Mao

**Affiliations:** ^1^Department of Computer Science and Technology, Shandong University of Finance and Economics, Jinan 250014, China; ^2^Shandong Provincial Key Laboratory of Digital Media Technology, Jinan 250014, China; ^3^Shandong China-U.S. Digital Media International Cooperation Research Center, Jinan 250014, China

## Abstract

Accurate segmentation of the tongue body is an important prerequisite for computer-aided tongue diagnosis. In general, the size and shape of the tongue are very different, the color of the tongue is similar to the surrounding tissue, the edge of the tongue is fuzzy, and some of the tongue is interfered by pathological details. The existing segmentation methods are often not ideal for tongue image processing. To solve these problems, this paper proposes a symmetry and edge-constrained level set model combined with the geometric features of the tongue for tongue segmentation. Based on the symmetry geometry of the tongue, a novel level set initialization method is proposed to improve the accuracy of subsequent model evolution. In order to increase the evolution force of the energy function, symmetry detection constraints are added to the evolution model. Combined with the latest convolution neural network, the edge probability input of the tongue image is obtained to guide the evolution of the edge stop function, so as to achieve accurate and automatic tongue segmentation. The experimental results show that the input tongue image is not subject to the external capturing facility or environment, and it is suitable for tongue segmentation under most realistic conditions. Qualitative and quantitative comparisons show that the proposed method is superior to the other methods in terms of robustness and accuracy.

## 1. Introduction

Tongue diagnosis is one of the important diagnostic methods of traditional Chinese medicine, while for a long time, tongue diagnosis relied on the doctor's clinical experiences by short-term visual observation, which causes the subjective and uncertain diagnosis results. With the development of image processing and machine learning technology, the research about intelligent assistant diagnosis of tongue manifestation in Chinese medicine has attracted more and more attention. Tongue segmentation from the background with teeth, lips, and face is the important step in the process of computer-aided tongue diagnosis and also an important premise to extract and analyze the color, texture, and morphology features of tongue quality and fur character. However, due to the limitation of the image acquisition process, the tongue with its surrounding tissue in the tongue image is similar in color and blurred of the outline; it is a challenge to propose an automatic, accurate, and universal tongue segmentation method.

The article "LSM-SEC: Tongue Segmentation by the Level Set Model with Symmetry and Edge Constraints" was published in 2021. Journal: Comput Intell Neurosci.

Tongue segmentation is also an image segmentation task. Image segmentation is a process of dividing an image into several homogenous regions that do not overlap each other. It is an important part of the image processing and is of great significance for image analysis, pattern recognition, and computer vision. From the classical image processing methods [1–3] to the deep learning [4–9], image segmentation has been widely concerned and applied. Traditional methods often focus on segmentation based on image features and variable models, and the level set model is one of the most representative methods of the active contour model. In 1987, the active contour models (ACM) were proposed by Kass et al. [10] firstly, which treated the image segmentation as an energy optimization problem and opened up a new view of image segmentation [10–13]. In recent years, the deep learning method can better perform automatic segmentation and can improve segmentation speed and robustness because of its excellent feature learning and representation ability [6–9]. SegNet [6] provides a full convolution network for pixel level image segmentation, while DFN [7] constructs a smooth network and a border network to form a discriminative feature network. LEDnet [9] adopts an asymmetric codec structure to solve the segmentation task in real-time scenes. These learning-based segmentation methods are widely used in various fields such as medical diagnosis [14].

In fact, in the process of tongue image acquisition, due to the influence of external conditions such as light and temperature, the tongue image is prone to the problems of tongue body position error and spot noise. And, due to the low-contrast characteristic of the tongue image, tongue segmentation is more difficult than conventional image segmentation. Since 1990s, many scholars have made relevant research studies on accurate tongue segmentation [15–22]. In the early stage of research, it is difficult to get accurate results only by using the underlying information of the image. Many subsequent methods improve the accuracy and robustness of segmentation. For example, Huang et al. [19] used the mean shift to smooth the edge and the maximum between-class variance method to classify the image and then merged the regions to extract the tongue. In [20], tongue extraction was based on color building blocks, and sparse representation was used to calculate pixel probability. The method based on deep learning can acquire more image features and has better performance. Huang et al. [21] proposed an automatic tongue image segmentation based on an enhanced full convolutional network. Qu et al. [22] proposed an image quality evaluation method based on brightness statistics to determine whether the input image needs to be segmented and used SegNet to train the tongue dataset. These methods avoid the complicated process of manually extracting features and have obvious advantages in segmentation performance.

The article "LSM-SEC: Tongue Segmentation by the Level Set Model with Symmetry and Edge Constraints" was published in 2021. Journal: Comput Intell Neurosci.

It is worth mentioning that the active contour model and some variants began to be applied in the field. For instance, Yang [23] presented a gradient vector active contour model based on the original tongue edge detection method and color gradient and obtained a good segmentation effect. In [24], the original tongue contour was obtained by extracting the ROI of the tongue and using the color similarity of the histogram, and then, the tongue segmentation combining region model and edge model were proposed. From the perspective of transforming the color space model, researchers proposed some effective algorithms based on color information [25–30].

However, it should be noted that the above algorithms usually have certain restrictions and requirements on the tongue image collection environment and the tongue image itself. Therefore, the results of tongue image segmentation with incorrect tongue body position and large noise influence are often not ideal. At the same time, there are other tissues such as peri lip in the image, and the color features of these parts are very close to the tongue itself, which results in the slow change of the gradient of the tongue edge. This leads to problems such as incomplete segmentation and boundary leakage in level set methods that rely on active contour models or gradient information to extract edges, and the accuracy of segmentation results is difficult to guarantee. Moreover, the active contour model is sensitive to the initial position; then, the adaptability is not satisfied.

In view of the above problems, we propose a symmetry and edge-constrained level set model for tongue segmentation. Different from the traditional level set model, the edge probability value is calculated using the latest convolutional neural network, and the obtained edge probability map is used as the gradient input of the level set. Considering the symmetry characteristics of the tongue, we add a symmetry detection constraint to the level set evolution model to test the symmetry feature of the zero level set contour. A novel level set initialization method is also proposed. It is proved by experiments that this method can complete automatic precise tongue segmentation suitable for most real situations.

The article "LSM-SEC: Tongue Segmentation by the Level Set Model with Symmetry and Edge Constraints" was published in 2021. Journal: Comput Intell Neurosci.

## 2. Related Work

Osher and Sethian [31, 32] proposed a level set method based on the important idea of fluid, which solved the problem that the topological structure is not easy to change during image segmentation. The level set method implicitly represents the closed active contour as a zero level set of a higher dimensional level set function and uses the curve evolution to locate the edge of the target. A lot of improvement work related to this appeared later. For example, Li et al. [33] proposed the distance regularized level set evolution (DRLSE) based on distance reinitialization in the process of level set evolution. Zhong et al. [34] proposed a level set method based on region consistency detection by considering the consistency of image region information and achieved good experimental results.

The main idea of the level set method is to regard the physical section moving with time *t* as the zero iso-surfaces of the level set function and transform the contour transformation of the *n*-dimensional surface into the evolution of the *n*+1 dimensional level set function; the boundary of it is expressed by the zero level set of the higher dimensional level set function. The active contour *C* is represented as a zero level set of the higher dimensional level set function *φ*(*x*, *y*, *t*), denoted as *C*(*t*)={(*x*, *y*)*|φ*(*x*, *y*, *t*)=0}. The purpose of the level set method is to make the zero level set *C* meet the partial differential equation of curve evolution:

(1) $$\begin{array}{c} \frac{\partial C}{\partial t}=V\left(k\right)N. \end{array}$$

For the above formula, the evolution equation of the zero level set *φ* under the velocity function *F* is

(2) $$\begin{array}{c} \frac{\partial \varphi }{\partial t}+F\left|\nabla \varphi \right|=0. \end{array}$$

The velocity function *F* depends on the image data and the level set function *φ*. In the image segmentation, *F* generally contains the curvature *k* of the evolution curve *C*. The curvature is calculated as follows:

(3) $$\begin{array}{c} k=\text{div}\left(\frac{\nabla \varphi }{\left|\nabla \varphi \right|}\right)=\frac{\varphi_{xx}\varphi_{y}^{2}-2\varphi_{x}\varphi_{y}\varphi_{xy}+\varphi_{yy}\varphi_{x}^{2}}{{\left(\varphi_{x}^{2}+\varphi_{y}^{2}\right)}^{3/2}}. \end{array}$$

If it is under the average curvature, the evolution equation can be written as

(4) $$\begin{array}{c} \frac{\partial \varphi }{\partial t}=\left|\nabla \varphi \right|\text{div}\left(\frac{\nabla \varphi }{\left|\nabla \varphi \right|}\right). \end{array}$$

One advantage of the level set method is that the calculation of curves and surfaces can be performed on a fixed Cartesian grid, and the evolution of the curve is independent of parameters. However, in the conventional level set methods, with the evolution of the curve, the level set function will no longer remain as the signed distance function. Therefore, it is necessary to periodically initialize the level set function to the signed distance function during the curve evolution. The process of reinitialization can affect the accuracy of the calculation, and it is time-consuming. To solve this problem, Li et al. added a distance regularization term to the conventional level set model and proposed a DRLSE [33] model without reinitialization.

The article "LSM-SEC: Tongue Segmentation by the Level Set Model with Symmetry and Edge Constraints" was published in 2021. Journal: Comput Intell Neurosci.

The energy function of the DRLSE model is as follows:

(5) $$\begin{array}{c} \varepsilon_{\text{DRLSE}}\left(\varphi \right)=\mu R_{p}\left(\varphi \right)+\lambda L\left(\varphi \right)+\alpha A\left(\varphi \right)=\mu \int_{\Omega }p\left(\left|\nabla \varphi \right|\right)\text{d}x+\lambda \int_{\Omega }g\delta \left(\varphi \right)\left|\nabla \varphi \right|\text{d}x+\alpha \int_{\Omega }gH\left(-\varphi \right)\text{d}x, \end{array}$$

where *μ*, *λ*,  and *α* are constant with positive values, representing the weight of each energy term.

The first term is a regularization term that constrains the deformation of the curve by guaranteeing the signed distance property |∇*φ*|=1. It is not necessary to reinitialize the level set function acyclically after adding the regularization term.

The second term is used to drive the zero level set to evolve towards the target edge. The function *g* is a boundary stop function based on the image gradient. Once the zero level set curve arrives at the target boundary, the energy function of the length term is the smallest.

The third term is the area term, which can accelerate the convergence of the zero level contour during the evolution of the level set. When initializing the level set, if the target is completely inside the initial curve, *α* should take a positive number to ensure that the curve converges inward; on the contrary, it should take the negative number.

The edge stop function *g* is defined as

(6) $$\begin{array}{c} g=\frac{1}{1+{\left|\nabla G_{\sigma }*I\right|}^{2}}, \end{array}$$

where *I* is the image to be segmented and *G*_*σ*_ is the standard deviation of the Gaussian filter.

According to the variational theory, in order to solve the gradient descent flow of energy functional, the following level set evolution equation is obtained as

(7) $$\begin{array}{c} \frac{\partial \varphi }{\partial t}=-\frac{\partial \varepsilon_{\text{DRLSE}}\left(\varphi \right)}{\partial \varphi }=\mu \text{div}\left(d_{p}\left(\left|\nabla \varphi \right|\right)\nabla \varphi \right)+\lambda \delta_{\varepsilon }\left(\varphi \right)\text{div}\left(g\frac{\nabla \varphi }{\left|\nabla \varphi \right|}\right)+\alpha g\delta_{\varepsilon }\left(\varphi \right), \end{array}$$

where the Heaviside function *H*_*ε*_*U*__(*x*) (see the third term in formula (5)) is used to divide the evolution region in the level set evolution, and the Dirac function *δ*_*ε*_*U*__(*x*) is the derivative function of the Heaviside function, which is used to constrain the evolution value. They are formulated by the following smooth functions:

(8) $$\begin{array}{c} H_{\varepsilon }\left(x\right)=\left\{\begin{array}{cc} \frac{1}{2}\left(1+\frac{x}{\varepsilon }+\frac{1}{\pi }\sin\left(\varepsilon \right)\right), & \left|x\right|\leq \varepsilon ,\\ 1, & x>\varepsilon ,\\ 0,x & x<-\varepsilon , \end{array}\right.\\ \delta_{\varepsilon }\left(x\right)=\left\{\begin{array}{cc} \frac{1}{2\varepsilon }\left(1+\cos\left(\frac{\pi x}{\varepsilon }\right)\right), & \left|x\right|\leq \varepsilon ,\\ 0, & \left|x\right|>\varepsilon . \end{array}\right. \end{array}$$

In recent years, the active contour model, level set, and some variants have been applied to tongue segmentation; Li [25] added the prior information of the difference between tongue and other parts in HSV color gamut to the level set model and proposed a new region-based bounded pressure function. Shi et al. [28] combined the geometric snake model with the parameterized GVFSnake [27] model and built the C2G2FSnake model, which improved the segmentation accuracy.

The article "LSM-SEC: Tongue Segmentation by the Level Set Model with Symmetry and Edge Constraints" was published in 2021. Journal: Comput Intell Neurosci.

## 3. The Proposed New Method

Due to the speciality of the pathological tongue and the limitation of image acquisition equipment, the difficulties of tongue segmentation are mainly reflected in the following aspects:

(1) The color of the tongue is similar to the surrounding tissues in the image background, so the color contrast is low. (2) The position of the tongue is not correct, and the spot noise is common in tongue segmentation. (3) The surface of the tongue has a thick coating or the tongue is cracked in the middle of the tongue. These factors lead to small differences in gradient values; then, the gradient map of the tongue is blurred. Therefore, the segmentation curve usually cannot be accurately stopped at the edge of the target contour, which greatly increases the difficulty of tongue segmentation.  Figure 1 shows the segmentation results of the DRLSE method for low-contrast, speckle noise, and thick coating images.

The level set method can calculate curves and surfaces on fixed Cartesian meshes and can deal with various topological changes as well, which is very suitable for medical image segmentation. As well known, the geometric characteristics of an image can clearly reflect the structural and content characteristics of the image and can prevent the image texture from being easily affected by interference factors such as light and noise. As the basic shape characteristic of an object, symmetry is ubiquitous in the nature, and the tongue as a part of the human body has the characteristics of mirror symmetry and rotation invariance. Therefore, the extraction of symmetry geometric features of the tongue image has a good guiding effect on tongue segmentation. Based on the above findings, the symmetry information is added to the level set model as a constraint by using the symmetry characteristics of the tongue image. At the same time, in recent years, the convolutional neural network has shown its unique advantages in complex or low-contrast image processing. Therefore, this paper combines the convolutional neural network model with the level set model, by taking the gradient map of neural network training as the gradient input of the level set to guide the curve evolution, and then proposes a symmetry and edge-constrained level set model for tongue segmentation.

The article "LSM-SEC: Tongue Segmentation by the Level Set Model with Symmetry and Edge Constraints" was published in 2021. Journal: Comput Intell Neurosci.

The principle of the symmetry detection constraint is that, during the process of level set segmentation, if the zero level set curve evolves to a weak gradient or strong noise, at that time, the zero level set function does not maintain symmetry; then, the constraints on the incomplete side of the segmentation and the energy will increase under the combined action of internal energy and external force of image symmetry. Conversely, if the zero level set function remains symmetrical during the segmentation process, the constraint term does not participate in the evolution process. Meanwhile, the evolution process of the level set function is to solve the DRLSE energy function of the minimized closed curve.

The initial contour is usually fixed to a rectangular area at an arbitrary position in traditional methods. In fact, the selection of the initial contour has a great impact on the segmentation results. Inappropriate position of the initial curve will cause the level set function to fall into a local minimum position. In this paper, we also extract the initial contour of the level set in a novel way. According to the characteristics of the constructed symmetry detection energy item, we first obtain the symmetry axis of the tongue body and set the initial contour curve as a circular region.

The key steps of the algorithm include the following: the convolution neural network is used to train the color tongue image, and the edge probability map is obtained as the gradient image input of the level set model. Then, we use the mirror symmetry of the tongue image to select the symmetry axis of the tongue automatically and take the symmetrical axis as the centre of the circle to get the initial contour curve located in the centre of the tongue. During the process of evolution, the evolutionary image and the gradient image are reflected and transformed, and the symmetry detection energy term is constructed to constrain the level set evolution. Finally, we use the variational method to solve the gradient descent flow of the energy function as to obtain the target boundary. The specific flow of the algorithm is shown in Figure 2.

The article "LSM-SEC: Tongue Segmentation by the Level Set Model with Symmetry and Edge Constraints" was published in 2021. Journal: Comput Intell Neurosci.

## 4. The Symmetry and Edge-Constrained Level Set Model for Tongue Segmentation

Compared with the traditional model, our improvements are as follows: adding the symmetry detection constraints, putting forward a symmetry and edge-constrained level set model, determining the symmetry axis of the tongue and changing the initial contour curve accordingly to match the functional characteristics of the symmetry constraint item, and combining the deep learning method to train the gradient input to improve edge accuracy. Next, the technical details will be described in the above order, not the order of the algorithm implementation steps.

### 4.1. Symmetry Detection Constraint

As mentioned above, the tongue has obvious symmetry; the symmetry detection constraint is used to detect the symmetry of level set function *φ* under the gradient image on both sides of the symmetry axis. The proposed detection constraint is based on a simple but important fact: if a plane geometry figure is approximately symmetric about the major axis, there must be a reflection transformation that minimizes the error of the transformed figure aligned with the original figure. Then, the difference between the energy of the DRLSE level set function and the energy after reflection transformation to the energy function is added as a symmetry detection constraint. The essence of the constraint is to evaluate the approximate symmetry of the target contour in the segmentation process.

Axis reflection transformation on the Euclidean plane and mirror reflection transformation in the Euclidean space are called reflection transformation. Reflection transformation is an important transformation in the Euclidean geometry. In this paper, the reflection transform is a horizontal mirror transform. Specifically, the symmetry axis of the image is used as the transformation axis to swap the pixels of the image. The original level set and the transformed level set in the evolution process are shown in Figure 3. The matrix *M* of the reflection transformation is expressed as

(9) $$\begin{array}{c} \frac{1}{A^{2}+B^{2}}\left[\begin{array}{ccc} B^{2}-A^{2} & -2AB & -2AC\\ -2AB & A^{2}-B^{2} & -2BC\\ 0 & 0 & 1 \end{array}\right], \end{array}$$

where *A*, *B*, and *C* are the coefficients of the general formula of the straight line *l*, and the calculation formulas of the coefficients *A*, *B*, and *C* are as follows:

(10) $$\begin{array}{c} \left\{\begin{array}{c} A=\left(y_{1}-y_{2}\right),\\ B=\left(x_{2}-x_{1}\right),\\ C=\left(x_{1}*y_{2}-x_{2}*y_{1}\right). \end{array}\right. \end{array}$$

In the evolution process of the level set function, if *Q*(*x*, *y*) is a point on the zero level set, the calculation formula of the new coordinate *Q*(*x*′, *y*′) after the reflection transformation with *l* as the symmetry axis is as follows:

(11) $$\begin{array}{c} Q^{\prime }=M*Q. \end{array}$$

If an image *I* is symmetrical, $\hat{I}$ is defined as a symmetrical complementary image of the source image, and the position of the pixels on $\hat{I}$ is derived from equation (11). The coordinates of point *Q*(*x*, *y*) for reflection transformation are as follows:

(12) $$\begin{array}{c} \left(\begin{array}{c} x^{\prime }\\ y^{\prime }\\ 1 \end{array}\right)=\frac{1}{A^{2}+B^{2}}\left(\begin{array}{ccc} B^{2}-A^{2} & -2AB & -2AC\\ -2AB & A^{2}-B^{2} & -2BC\\ 0 & 0 & 1 \end{array}\right)\left(\begin{array}{c} x\\ y\\ 1 \end{array}\right). \end{array}$$

For any given signed distance function, a transformed signed distance function that preserves shape invariance can be obtained by the above transformation. In the evolution process, *φ* is used to represent the priori shape, and the Heaviside function of *φ* in the gradient image is denoted as *H*_*ε*_(−*φ*)*g*. According to the above reflection transformation formula, the symmetric complementary term is ${\hat{H}}_{\varepsilon }\left(-\varphi \right)\hat{g}$. For solving the symmetric complementary term, the value of matrix *M* will be updated with the iteration of level set function *φ*. The definition of the symmetry detection constraint is shown in the formula:

(13) $$\begin{array}{c} S_{g}\left(\varphi \right)=\eta \int_{\Omega }{\left(H_{\varepsilon }\left(-\varphi \right)g-{\hat{H}}_{\varepsilon }\left(-\varphi \right)\hat{g}\right)}^{2}\text{d}x, \end{array}$$

where *η* is a positive number and *H*_*ε*_(−*φ*) is a Heavyside function of the level set *φ*.

The article "LSM-SEC: Tongue Segmentation by the Level Set Model with Symmetry and Edge Constraints" was published in 2021. Journal: Comput Intell Neurosci.

In image domain Ω, we measure the approximate symmetry of the target's own contour by the difference between the original level set function and the reflected transformed level set function. The computation on difference is completed by the symmetry detection constraint.

The energy function of the symmetry detection level set model is expressed as follows:

(14) $$\begin{array}{c} \varepsilon_{\text{SCT}-\text{DRLSE}}\left(\varphi \right)=\mu R_{P}\left(\varphi \right)+\lambda L_{g}\left(\varphi \right)+\alpha A_{g}\left(\varphi \right)+\eta S_{g}\left(\varphi \right)\\ =\int_{\Omega }p\left(\left|\nabla \varphi \right|\right)\text{d}x+\lambda \int_{\Omega }g\delta_{\varepsilon }\left(\varphi \right)\left|\nabla \varphi \right|\text{d}x+\alpha \int_{\Omega }gH_{\varepsilon }\left(-\varphi \right)+\eta \int_{\Omega }{\left(H_{\varepsilon }\left(-\varphi \right)g-{\hat{H}}_{\varepsilon }\left(-\varphi \right)\hat{g}\right)}^{2}\text{d}x, \end{array}$$

where *λ*, *α*,  and *η* are the coefficients of each energy term, the first three terms of the formula belong to the DRLSE model, and the last one is the symmetry detection constraint term (SCT).

The optimization of this energy function can be obtained with the following gradient flow descent method:

(15) $$\begin{array}{c} \frac{\partial \varphi }{\partial t}=-\frac{\partial \varepsilon_{\text{SCT}-\text{DRLSE}\left(\varphi \right)}}{\partial \varphi }=-\frac{\partial \varepsilon_{\text{DRLSE}\left(\varphi \right)}}{\partial \varphi }-\eta \frac{\partial S}{\partial \varphi }\\ =\mu \text{div}\left(d_{p}\left(\left|\nabla \varphi \right|\right)\nabla \varphi \right)+\lambda \delta_{\varepsilon }\left(\varphi \right)\text{div}\left(g\frac{\nabla \varphi }{\left|\nabla \varphi \right|}\right)+\alpha g\delta_{\varepsilon }\left(\varphi \right)+2\eta \delta_{\varepsilon }\left(\varphi \right)\left(H\left(\varphi \right)-H\left(\hat{\varphi }\right)\right). \end{array}$$

Obviously, the higher the symmetry of level set function *φ*, the smaller the value of SCT and the less the energy of constraints on evolution. If the image information is asymmetric, such as when the curve evolves to weak edges or tongue noise and tongue cracks, the symmetry of level set function *φ* decreases, and then, the value of SCT increases, which promotes the evolution of the side curve under the effect symmetry detection constraints.

A schematic diagram of LSM-SEC level set evolution is given in Figure 4.

### 4.2. Automatic Determination of Initial Contour

In the actual process of image acquisition, the tongue is usually captured in the middle of the image. Considering this prior knowledge, the symmetry axis from the tongue gradient image is first extracted, and it is used as the reflection transformation reference line of the symmetry detection constraint (SCT). Considering the feature of the symmetry detection constraint (SCT), in order to maintain the original image force of the level set function under the initial condition, we set the initial level set function as a circular contour fixed in the target area.

The article "LSM-SEC: Tongue Segmentation by the Level Set Model with Symmetry and Edge Constraints" was published in 2021. Journal: Comput Intell Neurosci.

The extraction of the symmetrical axis can be divided into two steps: fixed axis and direction, that is, determining the position of the symmetrical axis and the direction of the symmetrical axis. Since the centre of gravity of an axisymmetric figure must be on the symmetrical axis, the position of the symmetrical axis is determined by calculating the centre of gravity *w*_1_(*x*_1_, *y*_1_) of the gradient image:  

(16) $$\begin{array}{c} X_{1}=\frac{\sum P_{i}x_{i}}{\sum P_{i}},\\ Y_{1}=\frac{\sum P_{i}y_{i}}{\sum P_{i}}, \end{array}$$

where (*x*_*i*_, *y*_*i*_) is the coordinates of the pixel and *p*_*i*_ is the pixel values.

The corner point is generally considered to be the point at which the brightness of the image changes abruptly or the point at which the curvature of the edge curve is maximum. The Harris corner detection algorithm is used to find the potential tip point in the middle position of the tongue. The Harris corner detection [35] algorithm defines a corner as a point whose gray value can be greatly changed by micro offset in any direction. The Harris corner detection algorithm assumes that the pixel gray value of point (*x*, *y*) is *I*(*x*, *y*), and the change of gray intensity of each pixel (*x*, *y*) moving (*u*, *v*) in the image is expressed as a differential operator:

(17) $$\begin{array}{c} E_{\left(x,y\right)}=\sum_{u,v}w\left(u,v\right){\left|I\left(x+u,y+v\right)-I\left(u,v\right)\right|}^{2}, \end{array}$$

where *w*(*u*, *v*) is the coefficient of the filter window.

The rule of tracking the tip of the tongue with the Harris corner detector is searching for *k* pixels on the left and right sides of the middle position of the image data. For each current point projection to the *y*-axis, set the *y*-axis threshold and find its mean coordinate *w*_2_(*x*_2_, *y*_2_). Determine the axial direction by finding the position average of the potential tip point. The acquisition of the symmetry axis is shown in Figure 5.

It is known that the barycentric coordinates are *v*_1_(*x*_1_, *y*_1_) and the tongue tip coordinates are *v*_2_(*x*_2_, *y*_2_). According to the general equation *Ax*+*By*+*C*=0 of the straight line, a straight line equation that can obtain two points passing *v*_1_ and *v*_2_ can be expressed as

(18) $$\begin{array}{c} l:\left(y_{1}-y_{2}\right)*x+\left(x_{2}-x_{1}\right)*y+\left(x_{1}*y_{2}-x_{2}*y_{1}\right)=0. \end{array}$$

Taking the line *l* as the axis of symmetry, the point on the zero level set function is transformed.

The article "LSM-SEC: Tongue Segmentation by the Level Set Model with Symmetry and Edge Constraints" was published in 2021. Journal: Comput Intell Neurosci.

The initial contour of level set evolution is fixed in the target area, by choosing the axes of the symmetry axis. The initial contour shape is set as a circular region with the axes as the centre, which ensures that the symmetry detection constraint does not act on the level set function *φ* in the initial segmentation state and maintains the image force of the original evolution process.

With the source image *M* and symmetry axis *l*, the intersection of the line *l* and the source image *M* is denoted by (*x*_*a*_, *y*_*a*_), (*x*_*b*_, *y*_*b*_), and the calculation formula of the axis coordinate *O* of the symmetry axis is

(19) $$\begin{array}{c} O\left(X,Y\right)=\left(\frac{\left(x_{a}+x_{b}\right)}{2},\frac{\left(y_{a}+y_{b}\right)}{2}\right). \end{array}$$

In general, the initial level set function is set as the signed distance function (SDF), which is defined as follows:

(20) $$\begin{array}{c} \varphi \left(x,y\right)=\left\{\begin{array}{cc} -d\left(\left(x,y\right),C\right), & \left(x,y\right)\in \text{inside}\left(C\right),\\ 0, & \left(x,y\right)\in C,\\ +d\left(\left(x,y\right),C\right), & \left(x,y\right)\in \text{outside}\left(C\right). \end{array}\right. \end{array}$$

The signed distance function satisfies |∇*φ*|=1, where *d* is the Euclidean distance from the point (*x*, *y*) to the zero level set.

In this paper, the symbol distance function is defined as a circular initialization level set function with the axis *O* as the centre and *R* as the radius. The expression is as follows:

(21) $$\begin{array}{c} d\left(X,Y\right)=\sqrt{X^{2}+Y^{2}}-R. \end{array}$$

### 4.3. Gradient Image Based on Edge Probability Prior

From the definition of the boundary stopping function, one can see that the accuracy of the tongue gradient map is very important to the segmentation results. The traditional level set method directly calculates the partial derivative of the original image in the horizontal and vertical directions to obtain the gradient, but at the fuzzy boundary or the discrete edge, the segmentation result is limited with small gradient change of the target tongue.

Convolution neural networks (CNNs), as a kind of deep network, have been widely used in image processing and pattern recognition in recent years. The basic structure of a convolutional neural network generally includes a convolutional layer, pooling layer, and fully connected layer. Given by that the traditional CNN edge detection method only uses the features of the last convolutional layer as the output, many features and details are lost in the convolution process. Liu et al. [36] proposed an edge detector using a richer convolution feature (RCF). The RCF network makes full use of multiscale and multilevel information, combines all meaningful convolution features in a holistic manner to perform edge detection, and obtains a clear probability boundary. The network achieved the best detection results on the BSDS500 database.

The article "LSM-SEC: Tongue Segmentation by the Level Set Model with Symmetry and Edge Constraints" was published in 2021. Journal: Comput Intell Neurosci.

In this paper, the multilayer network structure features of the RCF network model are used to obtain the edge probability map, which is used as the gradient image input of the level set to guide the evolution of the edge stop function.

The RCF network model uses the characteristics of the multilayer network structure to obtain an edge probability map. RCF is based on the VGG16 network, which consists of five modules, alternating convolutional and pooled layers and three fully connected layers. The first two modules contain two subconvolution layers with the same parameters, and the last three modules contain three subconvolution layers with the same parameters. The subconvolution layer features of each module are added pixel by pixel using else layer, and the results are fused. Different scale features can be obtained by sampling under the maximum pooling layer.

Different from the traditional VGG16 network structure, the RCF replaces the pooled layer and the fully connected layer of the fifth module with a convolutional layer of size 1 × 1 so that the training result retains spatial information. RCF also proposes a new loss function for each module, avoiding the gradient disappearance problem during network training. The loss function is defined as follows:

(22) $$\begin{array}{c} l\left(X_{i};W\right)=\left\{\begin{array}{cc} \alpha \cdot \log\left(1-P\left(X_{i};W\right)\right), & \mathrm{if}\;y_{i}=0,\\ 0, & \mathrm{if}\;0<y_{i}\leq n,\\ \beta \cdot \log\;P\left(X_{i};W\right), & \text{otherwise}, \end{array}\right.\\ \text{in which }\alpha =\lambda \cdot \frac{\left|Y^{+}\right|}{\left|Y^{+}\right|+\left|Y^{-}\right|},\\ \beta =\frac{\left|Y^{-}\right|}{\left|Y^{+}\right|+\left|Y^{-}\right|}. \end{array}$$

*where Y*+ and *Y*− represent a positive sample set and a negative sample set, respectively. The superparameter *λ* is used to balance the positive and negative samples. *P*(*X*) is a standard sigmoid function. RCF uses the Caffe deep learning framework, the other parameters are the same as the Caffe model, and the training experiments were performed using the NVIDIA TITAN X GPU. The RCF network structure diagram is shown in Figure 6.

The edge probability map trained by the RCF network is used as the gradient image input of LSM-SEC, replacing the original gradient input in the edge stop function. The Gaussian filtering of the RCF gradient image is carried into equation (14), and the evolution of the edge curve is guided by iteratively calculating the edge stop function in the process of level set evolution. As shown in Figure 7, *a* is the original image and *b* is the tongue gradient image acquired by the RCF.

The article "LSM-SEC: Tongue Segmentation by the Level Set Model with Symmetry and Edge Constraints" was published in 2021. Journal: Comput Intell Neurosci.

## 5. Experimental Results and Analyses

In the experiment, the tongue image dataset contains 550 tongue images, part of which is from GitHub's open-source dataset, with a total of 300 tongue images; the other part is provided by the teachers of the University of traditional Chinese medicine, with a total of 250 tongue images. The images in the dataset are different in size, shape, angle, and position, but they all contain the complete tongue body, which is suitable for this experiment. Due to the need of the follow-up experiments, the tongue images were flipped, randomly cropped, rotated, and other operations were performed to expand the dataset, and finally, 1100 images were obtained. The “ground truth” of each tongue image is manually marked by experts. In this section, we will make qualitative and quantitative analysis of the experimental results.

The experimental environment of the algorithm is MATLAB R2010b; the machine system: win7; memory: 4 GB. In RCF training, the weight of the 1 × 1 conversion layer in stages 1–5 is subject to a zero-mean Gaussian distribution, the standard deviation is initialized to 0.01, and the deviation is initialized to 0. Because the dataset is relatively small, the ratio of training data and test data is 7 : 3. All parts of the neural network in this paper are completed by NVIDIA TITAN X GPU.

The parameters of the experiment are set as follows: the time step of the level set is Δ*t*=1, the regularization parameter is *ε*=1.5, the length penalty term parameter is *λ*=2, the weighted area term is *α*=−2, the distance regularization coefficient is *μ*=0.2, and the convolution calculation window size is *σ*=1. The above parameters all maintain the original DRLSE method parameter settings, and the symmetry detection constraints' parameter is *η*=1.

### 5.1. Qualitative Analysis

We compare the proposed method with three other classical methods, including distance rule level set evolution (DRLSE) method [33], maximal similarity-based region merging (MSRM) [37], automatic tongue image segmentation utilizing prior knowledge (C2G2FSnake) [28], and SegNet-based method proposed in [22].The results of tongue segmentation are shown in Figure 8. It can be analyzed that the MSRM method is not effective for most tongue segmentation, the contour curve is not completely consistent with the tongue boundary, and the segmentation accuracy is low. As shown in the third row (c) of Figure 8, the tongue and upper lip portions are not identified, and the thick coated tongue of the row (3) and column (e) differs greatly from the true boundary. It can be seen from the row (4) that SegNet can hardly distinguish the background around the tongue, especially in the row (4) and the columns (e) and (f), teeth and lips are not recognized. The edge of the DRLSE-divided tongue is smooth, but since the DRLSE method only uses the gradient information and does not combine high-level features such as color information, the result of segmentation between the low-contrast and low-gradient portions of the tip and the lip is poor. As shown in the low-contrast tongue images in columns (a) and (b) of row (5) of Figure 8, the DRLSE method does not accurately segment the portion of the tongue that is similar in color to the circumference of the lips. From the segmentation result of row (6), we can see that the C2G2FSnake method preserves the main contour of the tongue better, but this method still cannot solve the noise interference on the edge of the tongue, such as the thick coated tongue image of the fifth line. In addition, due to the low robustness of the C2G2FSnake tipping point finding method, these results in the segmentation extraction results are often not obtained during the segmentation process. In the experimental dataset, other results of the method of this paper are shown in Figure 9.

The article "LSM-SEC: Tongue Segmentation by the Level Set Model with Symmetry and Edge Constraints" was published in 2021. Journal: Comput Intell Neurosci.

Combining the experimental results of Figures 8 and 9, we can conclude that the edge of the target tongue extracted by the method is smooth and can effectively copy with the tongue crack of the pathological tongue, such as the third line (d) and (f) image above. At the same time, by observing the pictures in the second row (d) column and the fourth row (b) column, it can be noted that the method in this paper is insensitive to the spot noise appearing on the surface of the tongue, which solves the problem of spot segmentation caused by the DRLSE method. On the qualitative point of view, the LSM-SEC method is superior to the other three methods in processing low-contrast tongue images, which greatly improves the segmentation accuracy. The accuracy is partly due to the fact that the level set method is more suitable for the change of the tongue contour topology, and the gradient image input makes the segmentation result insensitive to the cracks and thick coating on the surface of the tongue, and the contour is more stable. On the contrary, the symmetry detection constraint enables the segmentation curve to maintain a good symmetry characteristic of the original tongue at a weak gradient. In a word, we can see from the results that our method is relatively universal and can extract accurate tongue from the surrounding environment.

The article "LSM-SEC: Tongue Segmentation by the Level Set Model with Symmetry and Edge Constraints" was published in 2021. Journal: Comput Intell Neurosci.

### 5.2. Quantitative Analysis

In order to quantitatively measure the segmentation performance of the proposed method, we use the reca, prec, IoU, and *F*1-measure indicators to compare and analyze the segmentation accuracy of the four methods. Prec, reca, and IoU are the precision, recall, and cross ratio, respectively, and *F*1-measure is the harmonic mean of the accuracy and recall. The accuracy of segmentation represents the proportion of the real target region in the segmentation result, and the recall ratio represents the proportion of the segmentation result in the real target region. *F*1-measure is the weighted harmonic average of accuracy and recall, while IOU is the intersection and parallelism ratio of the real area and segmentation area. The four indicators reflect the accuracy of the segmentation method, which are defined as follows:

(23) $$\begin{array}{c} P=\frac{\text{TP}}{\text{TP}+\text{FP}},\\ R=\frac{\text{TP}}{\text{TP}+\text{FN}},\\ F_{1}=\frac{2*PR}{P+R},\\ \text{IOU}=\frac{A_{a}\cap A_{b}}{A_{a}\cup A_{b}}. \end{array}$$

The variables *A*_*a*_ and *B*_*b*_ represent the segmentation results of the model and the divisions given by the medical experts. FP, FN, and TP are false positive volume fractions, false negative volume fractions, and true positive volume fractions, respectively, as defined below:

(24) $$\begin{array}{c} \text{TP}=\frac{A_{a}\cap A_{b}}{A_{b}},\\ \text{FN}=\frac{A_{b}-\left(A_{a}\cap A_{b}\right)}{A_{b}},\\ \text{FP}=\frac{A_{a}-\left(A_{a}\cap A_{b}\right)}{A_{b}}. \end{array}$$

The closer the values of prec, reca, IoU, and *F*1-measure are to 1, the better the segmentation results are. The average reca of LSM-SEC is 95.6%, the prec is 97.2%, the IOU is 93%, and the *F*1-measure is 96.3%. Refer to Table 1 for index values of other methods.

Figure 10 is a comparison of the index results of the four methods. The abscissa is the mean value of the indicators of reca, prec, IOU, and *F*1-measure from left to right. Through the quantitative analysis of the four indicators, it can be concluded that the LSM-SEC algorithm represented by the yellow column is superior to the other methods in the segmentation effect of the tongue. The proposed method achieves accurate segmentation results on all clinical tongue images and has high robustness. In the MATLAB experimental environment, the average processing time of each image in this algorithm is about 49.2 seconds.

## 6. Conclusions

As aforementioned, tongue segmentation is an important basic step in the informatization of tongue diagnosis in traditional Chinese medicine. In this paper, we first introduce a symmetry and edge-constrained level set model, which combines the latest neural network model and level set segmentation method to improve the gradient accuracy. With the symmetry constraint and adjustment of the initialization position, the proposed approach realizes intelligent segmentation. As the basic of the expert system, the symmetry and edge-constrained level set model for tongue segmentation can realize automatic tongue segmentation without manual intervention and achieve the goal of intellectualization. Finally, we provide detailed experimental tests. The experimental results demonstrate the segmentation accuracy and robustness of the proposed algorithm.

The article "LSM-SEC: Tongue Segmentation by the Level Set Model with Symmetry and Edge Constraints" was published in 2021. Journal: Comput Intell Neurosci.

Machine learning has been widely used in the medical field and plays an important role in disease diagnosis. In assisted tongue diagnosis, the method based on deep learning can achieve end-to-end tongue segmentation, which greatly simplifies the tedious steps of the traditional segmentation method and runs faster, with higher accuracy and better robustness. But different learning methods have different efficiency and segmentation accuracy. Different training samples and different size data will also affect the segmentation accuracy. Therefore, in the future research, we can improve the segmentation effect by improving the network structure and training strategy. At the same time, in view of the small dataset of the tongue image, few-shot learning is also considered as the research direction in the future.

## Figures and Tables

**Figure 1:** (a) Low-contrast tongue. (b) Speckle noise tongue. (c) Thick coating tongue.

**Figure 2:** Flowchart of symmetry and edge-constrained level set model for tongue segmentation.

**Figure 3:** Schematic diagram of horizontal set reflection transformation.

**Figure 4:** The behavior of level set evolution in the LSM-SEC: (a) the contour of the level set after 10 iterations, (b) the level set function after 10 iterations, (c) the contour of the level set after 80 iterations, (d) the level set function after 80 iterations, (e) the contour of the level set after 300 iterations, (f) the level set function after 300 iterations, (g) the contour of the level set after 600 iterations, and (h) the level set function after 600 iterations.

**Figure 5:** Center of gravity detection and corner detection.

**Figure 6:** RCF network structure diagram.

**Figure 7:** (a) Original image. (b) Gradient image.

**Figure 8:** Comparison of the results of tongue image segmentation method. Column (a)-(b) are seven types of tongue image. Row (1) is the original image, row (2) is the ground truth, and rows (3)–(7) are the segmentation results of MSRM, SegNet, DRLSE, C2G2FSnake, and our LSM-SEC, respectively.

The article "LSM-SEC: Tongue Segmentation by the Level Set Model with Symmetry and Edge Constraints" was published in 2021. Journal: Comput Intell Neurosci.

**Figure 9:** LSM-SEC segmentation result. Items (a), (c), and (e) are listed as real images, and items (b), (d), and (f) are listed as LSM-SEC segmentation results.

**Figure 10:** Comparison of tongue image segmentation results.

**Table 1:** Quantitative results.

	*F*-measure	IOU	Prec	Reca
MSRM	0.856	0.759	0.842	0.885
DRLSE	0.909	0.834	0.925	0.897
C2G2FSnake	0.899	0.820	0.899	0.904
SegNet	0.838	0.727	0.905	0.802
LSM-SEC	0.963	0.930	0.972	0.956

## Data Availability

In the experiment, the tongue image dataset contains 550 tongue images, part of which is from GitHub's open-source dataset, with a total of 300 tongue images: https://github.com/BioHit/TongeImageDataset; the other part is provided by the project collaborator of the University of Traditional Chinese Medicine, with a total of 250 tongue images. The images in the dataset are different in size, shape, angle, and position, but they all contain the complete tongue body, which is suitable for this experiment. Due to the need of the follow-up experiments, the tongue images were flipped, randomly cropped, rotated, and other operations were performed to expand the dataset, and finally, 1100 images were obtained. The “ground truth” of each tongue image is manually marked by experts in traditional Chinese medicine.
